# Epidemiological Characteristics and Drug Resistance of Fungemia in General Hospitals from 2010 to 2019

**DOI:** 10.1155/2021/2529171

**Published:** 2021-11-02

**Authors:** Yanling Bai, Zhigang Zheng, Ting Liu, Zhongqiang Yan, Mingmei Du, Hongwu Yao, Yunxi Liu, Jijiang Suo

**Affiliations:** ^1^Department of Disease Control and Prevention, The First Medical Center of Chinese PLA General Hospital, Beijing 100853, China; ^2^Fuxing Road Outpatient Department, Jingnan Medical District of Chinese PLA General Hospital, Fuxing Road No. 22, Beijing 100842, China; ^3^First Department of Health Care, The Second Medical Center & National Clinical Research Center for Geriatric Diseases, Chinese PLA General Hospital, Beijing 100853, China; ^4^Department of Disease Control and Prevention, The Second Medical Center & National Clinical Research Center for Geriatric Diseases, Chinese PLA General Hospital, Beijing 100853, China

## Abstract

**Objective:**

This study intends to analyze the data of fungemia in a large tertiary hospital from 2010 to 2019, and is aimed at understanding its epidemic characteristics and drug resistance.

**Methods:**

The “Hospital Infection Real-Time Monitoring System” was used to retrieve the case information of patients who were hospitalized for more than 48 hours from 2010 to 2019. The questionnaire was designed to collect patients' basic information, infection situation, drug resistance, and other related information. Statistical software was used for analysis.

**Results:**

The fungi detection rate was in the range of 0.19%~0.75% in ten years, the average rate was 0.29%, and the rate 0.2%~0.3% since 2013, which was lower than that from 2010 to 2012. Non-*Candida albicans* was the main fungus, accounting for 62.50%. The drug resistance of non-*C. albicans* was higher than that of *C. albicans*, among which *C. glabrata* had the highest resistance rate. Data analysis showed that the patients with more serious basic diseases, combined with infection of other sites, surgery, long hospital stay, combination of antibiotics, and invasive catheterization, were more likely to occur fungemia.

**Conclusion:**

We should pay more attention to the patients with high-risk factors of fungemia and focus on the drug resistance of non-*C. albicans*, choose the right antifungal drugs, so as to improve the level of diagnosis and treatment.

## 1. Introduction

In recent years, with the increasing use of immunosuppressive agents, broad-spectrum antibiotics, and biological agents, as well as the extensive development of traumatic diagnosis and treatment measures, the incidence of fungemia has been increasing [1]. Compared with bacterial infections, the primary manifestations of fungemia are not obvious, as well as the diagnosis, the mortality is higher, and the prognosis is even worse. The results of other studies showed that fungemia ranks the fourth in hospital-acquired bloodstream infection cases [2], and the infection rate increases year by year [3, 4]; the mortality can be as high as 50%-71% [5]. The types of antifungal drugs are limited, mainly including triazole, polyene, and echinomycin. Currently, fluconazole and amphotericin B are mostly used empirically in clinical practice, resulting in an increasingly serious problem of fluconazole resistance.

In 2009, the first new “*Candida auris*” was reported in Japan, which was resistant to all three classes of antifungal agents, known as “*super fungi*” [6]. So far, the drug resistance of fungal infection has been widely concerned. Up to now,“*C. auris*” has been found in more than 30 countries and regions around the world, including China. Fungemia, due to its high mortality and poor prognosis, has attracted enough attention in clinical practice; if the drug resistance is widespread, the consequences are unimaginable.

This paper retrospectively analyzed the data from 2010 to 2019 of a large general hospital in Beijing, China, which had nearly 4,000 beds and received more than 200,000 patients annually, to investigate the epidemiological characteristics and drug resistance of fungemia in the past 10 years, so as to provide reference for the prevention, control, and treatment of fungemia, as follows.

## 2. Materials and Methods

### 2.1. Materials

From January 1, 2010, to December 31, 2019, all patients met the inclusion and exclusion criteria in the medical, surgical, and intensive care units of the hospital. The diagnosis of fungemia was confirmed by professional physicians engaged in nosocomial infection control and clinicians according to the diagnostic criteria and clinical symptoms of patients. A total 680 cases of the fungi were detected, resulting in 615 fungemia in 598 patients. There were 378 males and 220 females, age ranging from 1 day to 94 years old, with an average age of 60.77 ± 20.025 years old. This study was approved by the Ethics Committee of the hospital with the approval number S2019-142-02.

*Inclusion criteria:* (1) blood samples submitted during hospitalization; (2) patients hospitalized for more than 48 hours; (3) complete case data.

*Exclusion criteria:* (1) patients with less than 48 hours of hospitalization; (2) complicated with community acquired bloodstream infection; (3) repeated strains of the same patient within 7 days; (4) blood culture results suspect contamination; (5) patients with missing data.

*Diagnostic criteria for fungemia*: the same fungus has been cultured from blood sample for twice or more; one blood culture was positive, and the same fungus was cultured from other parts of the body; one blood culture was positive, and the same fungal infection was confirmed by biopsy or autopsy specimens. Diagnostic criteria for concomitant bacteremia: positive bacterial blood culture before and after positive fungal culture.

The clinical diagnosis was combined with the “Diagnostic Criteria for Hospital Infection (Trial)"issued by the Ministry of Health of the People's Republic of China in 2001 [7], including fever greater than 38°C or hypothermia less than 36°C, accompanied by shivering, and combined with one of the following conditions: invasion of portal or migration lesions; symptoms of systemic poisoning; SBP of less than 12 kPa (90 mmHg) or more than 5.3 kPa (40 mmHg) below the original SBP.

*Diagnostic criteria for Catheter-Related Blood Stream Infection (CRBSI):* according to the 2011 CDC guidelines for the prevention of CRBSI [8], CRBSI refers to patients with endovascular catheter or removal of endovascular catheter within 48 hours of bacteremia or mycosis, accompanied by fever (>38°C), chills, or hypotension and other manifestations of infection. There is no other specific source of infection except for the vascular catheter. Laboratory microbiological examination showed that bacteria or fungi cultured in peripheral venous blood were positive, or pathogens of the same species with the same drug sensitivity results were cultured from both the catheter section and peripheral blood.

### 2.2. Methods

Through the “Hospital Infection Real-Time Monitoring System”, the case information of patients with positive blood culture for fungi during the study period was obtained, and the gender, age, basic disease, disease diagnosis, department, length of hospital stay, operation situation, date of fungemia, pathogen name, drug sensitivity results, time, and type of invasive catheterization and antibiotic prophylaxis and so on and so forth were registered in detail. The detection rate, drug resistance, and clinical distribution of fungemia were analyzed by statistical software.

### 2.3. Experimental Methods

Medical staff in the clinical department strictly followed aseptic operation when patients chills and have high fever, the venous blood samples were extracted for 8-10 mL and injected into the blood culture bottle for immediate examination. When catheter-related infection was suspected, the central venous blood and the contralateral peripheral venous blood were extracted at the same time or take the catheter tip which has been removed. Blood samples were cultured using Bact/Alert 3D 120 automatic blood culture instrument from Bio-Merieux, France, and its supporting aerobic and anaerobic flask containing neutralizing antibiotics, as well as BACTEC 9120 automatic blood culture instrument from BD, USA, and its supporting fungus culture flask. The Vitek 2-compact automatic bacterial identification system and associated fungal identification card (YST) provided by Biomerieux were used for bacterial identification. The ATB Fungus3 kit provided by Biomerieux was used for drug sensitivity test. The quality control strain was *Candida albicans* ATCC 14053.

### 2.4. Statistical Analysis

Differences in categorical variables were assessed using a Pearson *χ*^2^ test. SPSS version 19.0 was used for all statistical analyses. A two-tailed *P* value of <0.05 was considered to be statistically significant.

## 3. Results

### 3.1. Detection Rate of Fungi

From 2010 to 2019, 233189 blood culture samples from patients in internal medicine, surgery, and intensive care unit were detected, and 680 fungi were detected, with the detection rate of 0.29%. Among them, 512 cases were detected by venous blood, and 168 cases were detected by central venous catheter tip. The detection rate in 10 years was 0.19%-0.75%, with the highest detection rate in 2010 and the lowest detection rate in 2018. Since 2013, the detection rate of fungi has been maintained in the range of 0.2%~0.3%, which is lower than that of 2010~2012. See Table 1 for details.

### 3.2. Distribution of Fungi

Among the 680 fungal strains, 250 were *C. albicans*, accounting for 37.50%, and 430 were non-*C. albicans*, accounting for 62.50%, of which *C. parapsilosis* was the highest, accounting for 25.74%, followed by *C. tropicalis* and *C. glabrata*, accounting for 15.29% and 12.65%, respectively. There was no obvious trend in the distribution of the four fungi detected in recent 10 years. See Table 2 and Figure 1 for details.

### 3.3. Drug Sensitivity Analysis

The drug susceptibility testing (DST) was mainly carried out for Itraconazole, Fluconazole, Voriconazole, and Amphotericin B. The total resistance rate was 5.2%. The resistance rate to Itraconazole was the highest (7.9%), followed by Fluconazole (6.1%) and Voriconazole (3.1%); no resistance to amphotericin B was found. *C. albicans* had low drug resistance to all drug, and the highest resistance rate to Itraconazoleonly only as 1.5%. Among non-*C. albicans*, the drug resistance rate of *C. glabrata* to Voriconazole was the highest at 28.8%, and that of *C. tropicalis* to Voriconazole was the highest at 12.7%, and that of *C. parapsilosis* to Fluconazole was 4.8%. In 10 years, a total of 8 strains were found which were resistant to three kinds of antibiotics (Voriconazole, Fluconazole, and Itraconazole) and mediated to Amphotericin B, including 5 strains of *C. tropicalis*, 1 strain of *C. albicans*, 1 strain of *C. glabrata*, and 1 strain of *C. parapsilosis*. The distribution years were 1 strain in 2014, 3 strains in 2015, 2 strains in 2017, 1 strain in 2018, and 1 strain in 2019, respectively. See Table 3 for details.

### 3.4. Clinical Characteristics Description of Fungemia

There were 615 cases of fungemia in 598 patients; among them, 207 cases were CRBSI. The overall mortality rate was 19.90%. Male patients accounted for 63.21%; female patients accounted for 36.79%. The age of 60-79 years old was the most, accounting for 39.30%, and 68.73% of the patients were complicated with other site of infection. The top three departments were hepatobiliary surgery (including ICU) (18.23%), intensive care unit (10.87%), and respiratory medicine (8.7%). Surgical patients accounted for 63.38%. 89.80% of the patients had indwelling deep vein catheter, the average use time was 41.39 ± 57.415 days, 57.86% of the patients used ventilator, the average use time was 16.17 ± 40.502 days, 79.26% of the patients used indwelling urinary catheter, the average use time was 27.23 ± 52.993 days. 99.67% of the patients used antibiotics during hospitalization, and the combined antibiotics rate was 97.66%, the average antibiotic use days were 47.97 ± 56.098 days. The average hospitalization days were 66.26 ± 142.696 days. See Table 4 for details.

## 4. Discussion

*Candida* sp. is a conditional pathogen of human gastrointestinal tract, oral and vaginal mucosa, and epidermis. Under normal circumstances, even if the culture is positive in the host site, it cannot be considered as a pathogen, but the blood is a sterile part of the human body; once cultivated, it is significant. In recent years, it has been reported that the incidence of hospital-acquired fungemia has been on the rise, due to the widespread use of broad-spectrum antibacterial drugs, glucocorticoids, immunosuppressants, and chemotherapy drugs, as well as the development of multiple invasive diagnosis and treatment operations such as central venous catheterization and hemodialysis [9, 10]. In this study, we investigated the detection of fungi in blood culture from 2010 to 2019 and found that the detection rate did not increase, but decreased from 2013. The analysis found that the total number of blood culture samples was 11439 in 2010, rising to 21,794 in 2013, and to 30,153 in 2019, increasing by about three times. However, the total number of positives samples did not increase significantly, leading to a decrease in the detection rate. The reasons may be as follows: (1) with the development of medical technology, clinical emphasis has been placed on strengthening the submission of blood culture for examination. The number of submission for examination has been improved significantly, but the detection rate is lower. There may be excessive submission, invalid submission, or clinicians' lax grasp of symptoms and signs.(2) With the improvement of medical technology and antibiotic efficacy, the resistance of fungi has increased, but the detection rate may not increase significantly, and more large sample studies are needed to verify this conclusions.

In recent years, it has been reported that the increasing clinical application of azole-based antifungal drugs has led to a gradual increase in the incidence of non-*C. albicans* bacteremia [11, 12]. In our study, non-*C. albicans* accounted for 62.50%, which was higher than that of 50.00% in related studies [13], and the common non-*C. albicans* isolated from blood culture were *C. parapsilosis*, *C. tropicalis*, and *C. glabrata*, which were consistent with related studies [14]. *C. albicans* accounted for 37.50%, which was the most common fungi causing hospital-acquired fungemia [15, 16]. There was no increasing or decreasing trend in the analysis of the four main fungi detected in recent 10 years.

Drug susceptibility testing is an important means to guide clinical medication and monitor drug resistance. In this study, among non-*C. albicans*, *C. glabrata* had the highest drug resistance rate, and the drug resistance rates to Itraconazole, Fluconazole, and Voriconazole were 28.8%, 12.1%, and 3.8%, respectively, which were higher than the mediating rate and drug resistance rate of Candida smoothing to azole antifungal agents reported in related studies, which were both about 5% [17], which is similar to the report of Chinese Hospital Invasive Fungi Surveillance Network (CIF-NET) [18]. The highest resistance rate of *C. parapsilosis* to Fluconazole was 4.8%; the highest resistance rate of *C. tropicalis* to Itraconazole was 12.7%; but *C. albicans* had low drug resistance to all drug, and the highest resistance rate to Itraconazole only as 1.5%, which was consistent with the results of higher drug resistance of non-*C. albicans* reported by relevant studies [19]. In recent years, Amphotericin B-resistant fungi have been reported [18], but no drug-resistant strains have been found in this study.

A total of 8 strains were found to be resistant to three kinds of antifungal agents (Voriconazole, Fluconazole, and Itraconazole) and mediated to Amphotericin B, including 5 strains of *C. tropicalis*, 1 strain of *C. albicans,* 1 strain of *C. glabrata*, and 1 strain of *C. parapsilosis*. Among the 8 patients, there were 3 cases of hematopathy, 3 cases of abdominal surgery, 1 case of pediatric medicine, and 1 case of neurology care unit. Among them, 7 cases were complicated with fungal infection of other parts and were treated with antifungal drugs and indwelling vessels for a long time. 3 of them died. The remaining patient was hemopathy who was repeatedly hospitalized with multiple antibiotics. “*Candida auris*” is resistant to three kinds of commonly used antifungal drugs (including azoles, polyenes, and echinocandins) [20]. In this study, the susceptibility tests of Echinocandins has not been detected in our hospital, and the mass spectrometric method for “*Candida auris*” was not developed, so these 8 strains could not be identified as “*Candida auris*”; however, the results also reminded us to pay attention to the drug resistance of non-*C. albicans* and the emergence of “*Candida auris*.”

In this group of data, the incidence of fungemia in male patients is higher than that in females, and the age range is 60~79 years, which is consistent with the European research reports that among patients with fungemia, the infection rate in male patients is higher than that in females, and the difference is particularly significant over the age of 50 [21]. In our study, the mortality of patients with fungemia was 19.90%, which was lower than that reported at home and abroad 28.00% [22, 23], which was related to the lack of data due to the automatic discharge of some critical patients. Potential risk factors include hemodialysis, invasive therapy (such as central static catheter, urinary catheter, and mechanical ventilation), extensive gastrointestinal surgery, application of broad-spectrum antibiotics, multiple sites, or continuous colonization of Candida, which is consistent with the results reported in relevant studies [24, 25]. In this study, most of the fungemia were distributed in the surgery department (hepatobiliary surgery (including ICU) (18.23%), intensive care unit (10.87%), indicating that major surgery before admission to ICU or major surgery during admission to ICU (especially gastrointestinal surgery) and intestinal bacterial shift may be the risk factors for the occurrence of fungemia. This is consistent with the results of Chow et al. [26]. In addition, fungemia is also distributed in respiratory, gastroenterology, cardiology, and hematology departments, which suggest that the detection of fungemia should not be limited to some departments; doctors of all departments should pay attention to fungemia.

In conclusion, patients with fungemia have the characteristics of more basic diseases, severe illness, and high mortality, and the patients are distributed in a wide range of departments. Non-*C. albicans* have high resistance to antifungal drugs. Clinicians should pay enough attention to the patients with high-risk factors of fungemia, to detect the occurrence trend, strain distribution, and antifungal drug resistance, in order to choose reasonable antifungal drugs to improve the level of diagnosis and treatment of fungemia [27].

## Figures and Tables

**Figure 1:** Distribution map of four main fungi detected in blood culture from 2010 to 2019.

**Table 1:** The detection of fungi in blood culture from 2010 to 2019.

Year	No. of samples	No. of fungi	Rate of fungi %	Proportion of fungi %
2010	11439	86	0.75	12.65
2011	12226	82	0.67	12.06
2012	15734	66	0.42	9.71
2013	21794	44	0.20	6.47
2014	23300	63	0.27	9.26
2015	26721	59	0.22	8.68
2016	29996	72	0.24	10.59
2017	30330	83	0.27	12.21
2018	31496	59	0.19	8.68
2019	30153	66	0.22	9.71
Total	233189	680	0.29	100.00

**Table 2:** Detection of fungi in blood culture from 2010 to 2019.

Fungal pathogens	No. of fungi	Proportion%
***C. albicans***	255	37.50
***Non-C. albicans***	425	62.50
*Candida parapsilosis*	175	25.74
*Candida tropicalis*	104	15.29
*Candida glabrata*	86	12.65
*Candida krusei*	13	1.91
*Filamentous fungi*	11	1.62
*Ji Yemeng candida*	6	0.88
*Candida inconspicua*	4	0.59
*Aspergillus fumigatus*	2	0.29
*Trichosporon cutaneum*	1	0.15
*Candida lusitaniae*	1	0.15
*Simulon Candida*	1	0.15
*Nameless candida*	1	0.15
*Others*	20	2.94
*Total*	680	100.00

**Table 3:** The drug resistance analysis of fungi.

	Voriconazole			Fluconazole			Amphotericin B			Itraconazole		
	*S*	*R*	*I*	*S*	*R*	*I*	*S*	*R*	*I*	*S*	*R*	*I*
*Candida albicans*	128 (99.2)	1 (0.8)	0	157 (98.7)	2 (1.3)	0	0	0	129 (100)	125 (96.9)	2 (1.5)	2 (1.5)
*Candida parapsilosis*	91 (94.8)	2 (2.1)	2 (2.1)	111 (88.8)	6 (4.8)	8 (6.4)	2 (2.1)	0	94 (97.9)	86 (89.6)	1 (1.0)	/
*Candida tropicalis*	56 (88.9)	6 (9.5)	1 (1.6)	64 (87.7)	6 (8.2)	3 (4.1)	0	0	63 (100.0)	52 (82.5)	8 (12.7)	/
*Candida glabrata*	49 (94.2)	2 (3.8)	1 (1.9)	57 (86.4)	8 (12.1)	1 (1.5)	3 (5.8)	0	49 (94.2)	35 (67.3)	15 (28.8)	2 (3.8)
*Ji Yemeng candida*	2 (100.0)	/	0	4 (100.0)	/	0	0	0	2 (100.0)	2 (100.0)	0	0
*Candida krusei*	5 (100.0)	0	0	0	5 (100.0)	0	0	0	5 (100.0)	1 (20)	2 (40)	2 (40)
*Candida inconspicua*	2 (100.0)	/	0	1 (50.0)	/	1 (50.0)	0	/	2 (100.0)	2 (100.0)	/	0
*Candida lusitaniae*	1 (100.0)	/	0	1 (100.0)	/	0	0	/	1 (100.0)	1 (100.0)	/	0
*Trichosporon cutaneum*	/	/	/	/	/	1 (100.0)	/	/	/	/	/	/
*Total*	336 (95.2)	11 (3.1)	6 (1.7)	402 (90.3)	27 (6.1)	16 (3.6)	5 (1.4)	0	348 (98.6)	306 (96.7)	28 (7.9)	19 (5.4)

**Table 4:** Clinical characteristics of patients with fungemia.

Variables	Grouping, no (%). of cases
Gender	Male, 378 (63.21%); female, 220 (36.79%)
Age	≤18, 32 (5.35%); 18~59, 222 (37.12%); 60~79, 235 (39.30%); ≥80, 109 (18.23%)
Prognosis of disease	Death, 119 (19.90%); discharge, 477 (79.77%); other, 4 (0.67%)
Combined with other site infection	Yes, 411 (68.73%); no, 187 (31.27%)
Departments	Hepatobiliary surgery, 109 (18.23%); intensive care unit, 65 (10.87%); respiratory medicine, 52 (8.70%); gastroenterology, 48 (8.03%); cardiovascular medicine, 46 (7.69%); cardiovascular surgery, 41 (6.86%); general surgery department, 40 (6.69%); neurology department, 35 (5.85%); emergency department, 33 (5.52%); hematology department, 25 (4.18%); oncology department, 22 (3.68%); other, 82 (13.71%)
Operations	Yes, 379 (63.38%); no, 219 (36.62%)
Indwelling deep vein catheter	Yes, 537 (89.80%); no, 61 (10.20%)
Used ventilator	Yes, 346 (57.86%); no, 252 (42.14%)
Indwelling catheter	Yes, 474 (79.26%); no, 124 (20.74%)
Used antibiotics	Yes, 596 (99.67%); no, 2 (0.33%)
Combined antibiotic use	Yes, 584 (97.66%); no, 12 (2.01%); unused, 2 (0.33%)
Days of indwelling deep vein catheter	41.39 ± 57.415
Days of used ventilator	16.17 ± 40.502
Days of indwelling catheter	27.23 ± 52.993
Days of antibiotic use	47.97 ± 56.098
Inpatient days	66.26 ± 142.696

## Data Availability

This study only used the data from 2010 to 2019 for the purpose of analyzing the changes of fungus, which did not involve personal privacy and disputes. The data used to support the findings of this study are available from the author and corresponding author upon request.
